# Exploring the Feasibility of Virtually Delivered Auricular Point Acupressure in Self-Managing Chronic Pain: Qualitative Study

**DOI:** 10.1155/2022/8079691

**Published:** 2022-08-29

**Authors:** Jennifer Kawi, Chao Hsing Yeh, Nada Lukkahatai, Robin L. Hardwicke, Thomas Murphy, Paul J. Christo

**Affiliations:** ^1^University of Nevada, School of Nursing, Las Vegas, NV, USA; ^2^University of Texas Health Science Center at Houston Cizik School of Nursing, Houston, TX, USA; ^3^Johns Hopkins University School of Nursing, Baltimore, MD, USA; ^4^University of Texas Health Science Center, McGovern Medical School, Houston, TX, USA; ^5^Johns Hopkins University School of Medicine, Baltimore, MD, USA

## Abstract

**Background:**

Chronic pain remains highly prevalent. Current pharmacological and non-pharmacological strategies have not adequately managed chronic pain which has contributed to disability and high healthcare costs. With existing challenges in providing adequate pain care and access, we tested vAPA, a virtually delivered, self-management intervention using Auricular Point Acupressure (APA) by mobile app and virtual consultations (telehealth). Our key purpose was to evaluate the feasibility of the vAPA in self-managing chronic pain in preparation for a future randomized controlled trial.

**Methods:**

We conducted a descriptive, qualitative study evaluating our 4-week vAPA intervention among 18 participants. We used directed qualitative content analysis. *Results and Conclusion*. Participants perceived that vAPA was feasible (acceptable, useable, practical, and beneficial). In addition, the following themes were gathered: better control of pain, less use of pain medications, self-management and motivation in pain, and expectations for pain relief. Refinements were recommended for the app, content, and delivery to improve study interventions. Findings are relevant in moving forward to a future randomized controlled trial and for wider implementation in a pragmatic clinical trial.

## 1. Introduction

Chronic pain is a major public health problem with increasing prevalence and is the leading cause of disability in the United States and worldwide [1–7]. Chronic pain is described as having an “unpleasant sensory and emotional experience [8],” lasting beyond usual healing time, persisting constantly for at least three months or half of the days for the past 6 months [9]. Approximately 20% of American adults suffer from chronic pain and 8% of them are highly impacted and burdened with limitations in their activities of daily living [1]. As such, chronic pain is the second most common reason for healthcare visits in the United States [5, 10], resulting in over $635 billion in medical care costs, loss of productivity related to disability, and lost wages [9]. Globally, 1 in 10 individuals suffer from chronic pain, leading to high healthcare needs, costs, and great societal burden [11].

Despite multiple pharmacotherapy and non-pharmacological modalities used to address chronic pain, inadequate management persists, contributing to the overutilization of healthcare resources with poor patient outcomes [12–14]. Pain management is an international basic human right [11] and the Institute of Medicine has recommended guidelines for non-pharmacological, self-management strategies to manage pain [9]; however, utilization of these strategies in clinical practice has been challenging and access to pain care continues to be limited [15]. The salient need for better pain management measures persists.

This study focuses on the use of Auricular Point Acupressure (APA) to assist patients in the self-management of their pain. APA is based on the principles of acupuncture which is a non-pharmacological modality supported with significant evidence in managing pain effectively, and hence has been recommended by current guidelines [15, 16].

With the Coronavirus-19 pandemic, the burden suffered by patients with chronic pain has been magnified [17] as the availability of pain treatments is limited from fewer in-person visits, thereby delaying adequate access to care [18]. Therefore, we conducted a pilot study to evaluate virtually delivered APA (vAPA). This qualitative research was done in the context of our pilot study with an overall goal to improve our intervention for a future randomized controlled trial (RCT). We were guided by the recommendations from O'Cathain and colleagues in maximizing the value of qualitative research in feasibility studies to prepare for an RCT [19]. Hence, our *overall purpose* was to *explore the feasibility of vAPA in the self-management of chronic pain.* The *overarching research question* was as follows: is vAPA feasible in self-managing chronic pain. The specific follow-up questions were related to key domains to evaluate feasibility such as perceived acceptability, usability, practicality, and benefits of vAPA [20, 21].

### 1.1. Background

Pharmacologic therapy such as analgesics—especially opioids—are the most common treatments used by patients for chronic pain; however, excessive and inappropriate opioid use has resulted in the current opioid epidemic [22–24]. Even other analgesics, such as nonsteroidal anti-inflammatory drugs, can potentially cause adverse effects such as renal insufficiency, gastrointestinal bleeding, hypertension, or congestive heart failure [22].

Non-pharmacologic modalities are recommended in guidelines but these have barriers to implementation, including limited access and availability, lack of insurance coverage, low reimbursement, high costs, limited capacity, and more time for required visits, among others [9, 15]. Even acupuncture, which is now included as one of the non-pharmacological modalities in pain management guidelines, has barriers to widespread implementation. Acupuncture involves complex provider assessment and individual treatment by trained providers (300 hours required for physicians or 1,800 hours of acupuncture training from an accredited school); its implementation is also limited due to labor intensity [25], inadequate insurance coverage [26, 27], a relative dearth of acupuncturists, and geographic inaccessibility [28].

Less accessibility and availability as well as the higher costs associated with certain pain treatment modalities present an excellent opportunity for APA in self-managing chronic pain. APA was derived from traditional Oriental Medicine's auricular acupuncture, developed into modern science in the 1980s by Paul Nogier, MD [29–31]. Dr. Nogier mapped a somatotopic representation of the human body onto the ear. Specific points on the ear (acupoints) correspond to specific organs and areas of the body and by stimulating these ear points, symptomatic parts of the body can be treated. For systematic diagnosis, locations of ear points corresponding to the symptomatic body part is confirmed by electrodermal responses (i.e., an electrical point finder or a small non-invasive probe) [32, 33]. Once the ear points are identified, acupuncture-like stimulations are introduced into these points, classically with the use of needles, electrically [33, 34], or with APA using pellets or Vaccaria seeds in a non-invasive manner [35]. Vaccaria seeds are natural, non-toxic botanical seeds of no medicinal value that is used in auricular acupressure. These seeds are applied to appropriate ear points; patients stimulate these ear points at least three times a day for three minutes each time, and any time during the day when they need to reduce pain. The underlying theory of auricular acupuncture posits that nerves in the outer ear correspond to specific areas of the brain, and that these areas have a reflex connection with specific parts of the body [33, 34]. The treatment of ear points can stimulate the brain to correct its pathological reflex centers [36], change levels of serum pro- and anti-inflammatory cytokines [37–40], and induce reflex reactions in the body to relieve body pathology [29, 34, 41].

Our interdisciplinary team has conducted several trials and accumulated significant evidence for chronic pain reduction using APA compared to sham APA. Our team demonstrated the following: (1) significant rapid and sustained effects on pain-related outcomes—APA resulted in rapid pain relief (≥38% three minutes post-APA [42, 43]) with >44% pain relief and >28% improved physical function at follow-up after 4 weeks of APA [35, 44–49]; (2) reduced use of pain medications—after 4 weeks of APA, ≥60% of participants reported less use of pain medications [35, 50]; (3) similar effectiveness between interventionist-administered vs. self-administered APA—we developed a self-guided, mobile-enabled APA application (app) to allow patients to self-administer APA[51]. After 4 weeks, 26 users showed an average reduction of 46% in pain intensity and 31% in pain interference [51]; and (4) successful integration of APA into a major healthcare system in real-world clinical practice [43, 52]—patients who received APA by trained nurses achieved 71% pain reduction post-48 hours of APA [43]. APA is now included in the electronic medical records of this major healthcare system in eastern US as one of the treatments for pain.

To further advance APA and prepare it for widespread dissemination—especially when in-person healthcare visits are limited—we developed and piloted our *vAPA intervention*. vAPA is a virtually delivered APA, leveraging technology using our tested mobile-enabled app featuring APA videos and supplemented with secured, remote video conferencing by Zoom. Participants received study instructions and were sent an APA kit containing a probe (used to find ear points) and seeds for placement along the ear points (about 2 mm in diameter) with pre-cut, waterproof tape used to secure the seeds (about 6 mm^2^) on their specific ear points. They were also given access to our app which provided detailed instructions, ear graphic images, and steps for finding ear points specific to their pain complaint through 2 short (5 minutes each) videos. Participants were then instructed to self-administer APA to manage their chronic pain for four weeks. During the first week of APA use, participants were advised to e-mail photographs of their ears showing their seed placements. A virtual session was scheduled individually to conduct sessions similar to telehealth and the following were performed systematically during this session: (1) review of ear photographs with ear point readjustments performed as needed especially considering current pain levels (inaccurate placement will not reduce pain), and further ear graphic images were provided to help with proper placement; (2) response to any questions from participants related to the intervention and their chronic pain; and (3) self-management support to facilitate participant capabilities and motivation to become active participants in their pain care [53, 54]. For data collection, we measured pain-related outcomes, analgesic use, and APA adherence. Time points included baseline (pre-intervention), immediate post 4-week intervention, and 1-month post completion. We then conducted interviews virtually at the last time point (1-month post completion). This manuscript describes the results of the interview findings.

In conducting this pilot study on vAPA, it was very important to conduct qualitative research to evaluate our intervention content and delivery, trial design and study processes, and outcomes. In doing so, the guidelines put forth by O'Cathain and colleagues were found useful and the best fitting to allow us to understand how our participants perceived vAPA in significant domains related to feasibility such as acceptability, usability, practicality, and perceived benefits. These were operationally defined and adapted for use in this study as follows: [20, 21] (1) *acceptability* (satisfaction, what participants like about the intervention, and their intent to continue); (2) *usability and implementation* (participant engagement and any changes or recommendations to the intervention); (3) *practicality* (cost and ability to carry out the intervention); and (4) *perceived benefits* (improvement in pain and related outcomes). These domains in evaluating feasibility were found to be the best addressed in a qualitative study [19].

Based on O'Cathain and colleagues [19, 55, 56], conducting this qualitative research allowed us to improve our planned intervention for refinement, explore possible challenges, and facilitate prospect optimization of the intervention in a future RCT. This process is important allowing for necessary changes with significant implications to inform a robust RCT. This qualitative research, therefore is placed within an evaluative framework [56, 57] for effective refinement of the vAPA.

## 2. Methods

### 2.1. Design

This is a descriptive, qualitative study focusing on the feasibility of vAPA. This qualitative research was conducted during piloting of the vAPA. We used the Consolidated Criteria for Reporting Qualitative Research checklist as a guide in reporting this study [58]. Quantitative findings were published in a separate manuscript [59]; this was submitted separately for publication due to the large amount of data gathered.

In conducting this qualitative research, we were guided by the recommended key steps from O'Cathain and colleagues: [19] (1) we identified the feasibility questions related to our pilot study for our vAPA intervention, (2) we selected the appropriate design and methods to address these questions, (3) we implemented our pilot study and conducted data collection while analyzing our qualitative data in an iterative and dynamic process, (4) we worked as a team throughout, and (5) we reported our findings, then, progressed to refining our intervention toward a future RCT for vAPA. These key steps provided clear guidance for applying qualitative research in a feasibility study prior to undertaking an RCT with the goal of improving the intervention for a full trial.

Three researchers (CY, NL, JK) conducted the interviews after conferring on the interview questions and process in order to facilitate consistency. These researchers worked with the larger team conducting the pilot study to have an adequate understanding of the overall study but independent enough so that the participants could offer honest feedback in the interview sessions. Two of these researchers are PhD-prepared faculty members and 1 is a PhD student—all with background, knowledge, and training in qualitative research.

### 2.2. Participants and Study Setting

Inclusion criteria were as follows: (1) 18 years or older, (2) pain that has persisted for at least 3 months or at least half of the days in the past 6 months, (3) average pain intensity ≥4 on a 11-point numerical pain scale in the previous week, (4) able to apply pressure to taped seeds on their ear points, and (5) access to a mobile device to be able to download our app and participate in our virtual session. Patients with the following were excluded: (1) malignant or autoimmune diseases, (2) known acute compression fractures, (3) use of some hearing aids that may obstruct placement of seeds on specified ear points, and (4) allergy to tape. Using purposing sampling, we received 31 referrals from healthcare providers at Johns Hopkins Medicine and 55 inquiries from individuals at different states who learned about our study from our advertisements. Fifty-six participants were excluded for various reasons (e.g., not meeting the inclusion criteria, changed their mind, unable to commit to study). Of the 30 remaining who were enrolled in this study, two dropped out because of new medical conditions unrelated to APA; one dropped out because of a very busy schedule, and two failed to schedule their post-intervention visit. Consequently, 25 participants completed this study (83% retention rate). The study setting was virtual; all research activities were completed remotely. The participants expressed a great interest given the remote nature of the study which facilitated recruitment.

### 2.3. Procedures

We received Institutional Review Board approval (IRB00158622) for our pilot study. Our participants completed their informed consents and emailed these to us through a secure university server. Data collection included conducting semi-structured interviews using pre-determined, open-ended questions relating to the feasibility of the vAPA. Interviews were used for data collection to better understand and explore participant experiences directed on the feasibility of the vAPA in self-managing their pain, addressing our overall study purpose. The study enrollment occurred between June and July 2020; data analyses were completed in November 2020. All authors communicated prior to the interviews to facilitate consistency in the interview guide and study processes. During these communications, the authors refined the interview guide to best reflect the overarching purpose of this qualitative research in evaluating the feasibility of the APA. The authors also communicated throughout the interview schedules as data were gathered and analyzed to further refine the questions. For example, evolving themes on having “better control of pain ” and “expectations for pain relief” were consistently communicated by participants from the initial interview questions regarding perceived benefits of the vAPA so these themes were further explored with the participants moving forward. This reflects the iterative and dynamic data collection and analyses of this qualitative study resulting in the emergence of important questions and production of subsequent data.

The in-depth interviews ranged from 30 to 60 minutes and were conducted 1 month after completing the vAPA intervention. Participants were interviewed based on their availability in a private setting of their choice. Secured interviews were video-recorded remotely with audio transcription. The recordings were kept confidential and secure in a university server with log-in information required, available only to the researchers involved in this study. Transcribed data, field notes, photographs, audit trails, and all participant-related information were deidentified and stored in password-protected computers.

### 2.4. Data Analyses

Data analyses were conducted using a deductive approach through qualitative content analysis. Content analysis is the most appropriate for exploratory studies to obtain answers needed for the identified overarching research questions [60]. Specifically, directed qualitative content analysis was conducted because of the need for a more structured process compared to a conventional approach for exploring the feasibility of the vAPA [61]. In this directed process, key feasibility domains were used for initial coding of the data into categories. These initial codings included acceptability, usability, practicality, and benefits [20, 21]. Operational definitions for each category were described previously. In reviewing various feasibility studies as well as current practices and guidelines [20, 21], it has been recommended that acceptability [20, 21], usability [20, 21], practicality [20, 21], and benefits [20, 21] be the important, key, and consistent foci necessary in the design and implementation of feasibility studies toward evidence-based interventions.

Four researchers immersed themselves in the data with repeated review of information and field notes. To help discern patterns that were systematic, data were organized into a table matrix based on the predetermined study questions and then coded manually based on the established categories. As data analyses continued throughout the interview processes, additional categories were formulated, refining the initial coding scheme. Subsequently, emerging themes resulted with continued checking and reverse process, gathering direct quotes from participant interviews supporting emerging themes. Any differences between the authors in these directed content analysis processes were resolved through discussions, and an audit trail was documented to record coding schemes and facilitate intercoder reliability. For example, it was deemed equally important to ask about any dislikes (other than what participants liked about the intervention or acceptability) and any negative impact (apart from perceived benefits). Dislikes and negative impacts were then categorized under “*Potential Barriers*” because the feedback related to these topics was not well-fitting under the four feasibility domains (see Table 1 for sample participant responses within each category).

Transcripts of the interviews were not returned to participants but member checking was conducted at the end of each interview, summarizing information gathered for accuracy or credibility and trustworthiness. A summary of the findings was further shared with 2 participants who expressed availability for review and subsequently agreed with the findings. No additional feedback or changes were received.

Throughout the study, the researchers practiced reflexivity (e.g., jotting notes and thoughts during an interview, reflecting after an interview and during transcription and data analysis). One of the research team members is a Master of Auricular Medicine, all others were trained or well-informed about APA. These knowledge and skills facilitated participant learning of APA, particularly in finding accurate ear points. However, reflexivity was practiced by the research team to minimize introducing bias, and enhance rigor and credibility [62].

## 3. Results

### 3.1. Characteristics of Participants

Twenty-five participants enrolled in the study. Three did not respond during the intervention phase, three decided to drop out because they felt that the intervention did not work, and one did not complete the interview due to a family emergency. A total of 18 participants completed our study. This number is considered appropriate for qualitative research in feasibility studies, where 5–20 are adequate, with up to 20 being able to identify about 95% of relevant data [19]. Participants were recruited through healthcare providers and self-referrals until emerging analyses showed no new knowledge was obtained, sufficient data were achieved, and data saturation was reached.

Table 2 presents the demographic characteristics of the participants (*n* = 18) who completed the study including the post-intervention interviews. The mean age of the participants was 52.39 (SD = 18.16) with a majority older than 50 years (*n* = 11, 61%) and most of them were women (*n* = 13, 72%). Approximately 56% (*n* = 10) took prescribed pain medications and 61% (*n* = 11) took over-the-counter pain medications. Some of the participants' prescribed medications commonly included opioids, adjuvant analgesics, and other agents including neuropathic medications, muscle relaxants, nonsteroidal anti-inflammatory agents (prescription dose), sleep aids, and benzodiazepines.

### 3.2. Major Themes

Based on the coding of our participant data with sample information in Table 1, we derived five themes: the overall major theme was that the *vAPA was feasible*. Other themes were: *better control of pain, less use of pain medications, self-management and motivation in pain, and expectations for pain relief* (see Table 3).

#### 3.2.1. vAPA Is Feasible

Based on participant responses, the overall major theme obtained was that vAPA is feasible. Several participant responses were noted in Table 1 that reflect acceptability, usability, practicality, and perceived benefits of the vAPA. Further, one participant stated overall, “the program is well organized and the staff members are helpful. ” Another participant stated, “I believe your team is doing a fantastic job in helping selflessly, by teaching and coaching patients this valuable technique. Thank you and keep up your altruistic work. ” There were also potential barriers particularly in initially locating ear points. Although all participants were able to successfully locate ear points accurately, two had initial challenges that were assisted with an additional virtual session, ear photos, and ear graphics pointing to precise locations. Participant responses on barriers to the treatment will serve to help improve the intervention. Importantly, no side effects nor adverse effects were noted.

#### 3.2.2. Better Control of Pain

It is clear that the participants perceived benefits from the intervention. For instance, the benefits included, among others, pain relief or reduction, improved sleep, reduced anxiety, and that the APA had meditative effects. Pain relief also appeared to include improvement of neuropathic symptoms such as tingling and numbness. Apart from these perceived benefits and specific to this theme, participants mentioned “control of pain” that they experienced with the APA as a highly recurring experience. The intervention was something they felt they could implement any time they were in pain and consequently felt reduced pain levels based on greater control over the treatment. One participant stated, “I like the fact that I feel I am in control of managing my pain. ” Another participant realized after the virtual session that he could press his ear points more frequently anytime he needed it for pain reduction. This feature of APA was reinforced during his virtual session, which resulted in better control of his pain.

#### 3.2.3. Less Use of Pain Medications

Because the participants experienced pain relief or reduction from the intervention, they consequently used their analgesics with less frequency. This is significant because the majority of the participants took pain medications, both prescribed and over-the-counter. Others who used some natural remedies or non-pharmacological modalities also needed less of these after incorporating APA. One participant mentioned that she did not need to go and seek pain relief from a healthcare provider during the study.

#### 3.2.4. Self-Management and Motivation in Pain

Many participants felt that personal motivation was important in being able to self-manage their pain. For example, if they actually used the APA to help with their pain, participated in the intervention, the experience of pain relief motivated them to continue further in using APA to self-manage their pain. One participant quoted a saying, “You get what you inspect, not what you expect. ” To achieve the best results in pain relief, participants were motivated to self-manage their pain, gave themselves the opportunity to try something new and different such as APA, engaged with the intervention, and subsequently experienced pain relief.

#### 3.2.5. Expectations for Pain Relief

Many participants were realistic about their expectations of pain relief. Even during instances when their pain did not reach zero, many participants were delighted that the APA treatment provided pain reduction, regardless of the amount of relief. Some were happy with a single point reduction of pain from their usual pain level on a scale of 0 to 10. Others were pleasantly surprised with the amount of significant pain relief they received, experiencing a substantial drop in their pain level. For example, a participant felt that her expectations for pain relief were met with her well-diminished pain so she “did not have to take pain killers around the clock” because APA significantly decreased her pain level.

## 4. Discussion

The qualitative approach conducted in this study is appropriate in feasibility and pilot studies and highly relevant for informing the research team, facilitating necessary changes toward improving the intervention prior to the conduct of an RCT [19]. Given all participant responses with examples noted in Table 1, we found that vAPA was feasible as a self-management tool for managing chronic pain. Participants found the intervention to be acceptable, useable, practical, and beneficial for their chronic pain and other related symptoms (e.g., numbness, tingling, anxiety, lack of sleep). Proceeding with an RCT would be the next logical step.

Exploring other participant themes, we also found that vAPA resulted in better control of chronic pain with easy access to this intervention whenever the need arises. Consequently, participants used fewer pain medications. This highlights an important potential future application of APA directed to decreasing unnecessary healthcare utilization and positively reducing current exorbitant healthcare costs associated with chronic pain [9]. Self-management of pain was also another important theme and key motivating factor for the participants to continue using APA. Self-management can influence the sustainability of APA for future use; patients implement interventions that are not only accessible but also interventions that they find beneficial, useful, and have immediate positive impact. In effect, patients become motivated and assume a more active role in self-managing their pain. It has been well documented that patients with chronic pain who actively engage in their own treatment achieve superior outcomes compared to those who take a passive approach [63, 64]. We also found that although there was some variability as to participants' pain relief expectations, many felt that even a single point drop in their usual pain level was valuable. This represents a significant finding for an intervention that is easily accessible and works immediately. Method triangulation [65] was performed to evaluate consistency of findings and enhance validity. Our quantitative findings [59] also showed reduced pain intensity among our participants.

In evaluating vAPA and assessing its ability to be scaled-up for widespread implementation and further testing, identifying potential barriers was necessary. These provided key opportunities and lessons learned for future studies to help address these barriers. For example, to assist in accurately locating ear points and securing the seeds, future intervention refinement will include the following: shorter, succinct, but additional graphic videos specific to each area of body pain with larger diagrams, larger fonts, closed captioning, and detailed instructions for better understanding and clearer demonstration of APA while maximizing its use as a self-guided tool to manage pain. The videos will reinforce the use of APA by recommending that patients press on the ear points anytime that pain recurs. This would be in addition to the minimum recommended APA practice of three times a day for three minutes each time. Additional virtual sessions may be necessary to address any questions and some may need another person to help secure the seeds to the proper ear point and minimize the seeds from falling off. We also found that some participants complained about the soreness on their ear points with the APA. There is ear soreness related to APA treatment because identifying the appropriate ear acupoints (site for acupressure stimulation) produces some initial discomfort. However, this soreness gradually disappears when body pain intensity improves [32, 66]. Thus, it is important to advise participants about this potential discomfort when they first receive APA treatment. Additionally, some participants experienced itching due to the tapes used to adhere the seeds to the ear points, indicating potential sensitivity or allergy to the tapes. Thus, a better adherent (i.e., non-allergenic tapes) should be used in future studies.

Additional refinements based on participant feedback include developing a website with educational videos including tips and Q & As, making the APA app web-enabled for easy viewing and accessibility on a computer or tablet, and using a skills checklist as a self-evaluation tool to ensure that all APA procedural steps are completed for the best results. These refinements will aid in facilitating adequate access to effective pain interventions even beyond the current pandemic given the existing challenges in accessing pain treatments and prevailing pain care disparities [67–69].

### 4.1. Implications

Significant implications related to the refinement of the vAPA intervention were discussed. Other important implications pertain to study recruitment and retention. Recruitment in this study was facilitated by its virtual delivery and retention was not difficult especially due to participant's perceived benefits from vAPA. Further strategies could include use of motivationally tailored messages to promote adherence, an individualized dashboard with each participant's own study outcomes for self-monitoring, participant video vignettes and discussion board to allow for networking and social engagement, and study newsletters to keep participants well-informed throughout the study. These enhancements are all important moving forward to an RCT and larger implementation by means of a pragmatic clinical trial.

The implications of this study can also lead to increasing training of APA among healthcare providers, community partners, interested patients, and other individuals for broader application to the general population. Education on the value of non-pharmacological, self-managed interventions among various stakeholders can help facilitate a significant paradigm shift in pain management interventions that are useful and less costly. Policy implications are important toward eventually covering APA in health insurances for better access to pain control for all patients with chronic pain and help address pain care disparities.

## 5. Limitations

This qualitative study highlighted the feasibility of vAPA which is important toward evaluating its utility toward a future RCT and further testing in a larger population of patients. However, there were limitations. Purposive sampling limits representativeness but the virtual nature of this study allowed us to recruit with a wider reach. In conducting the interviews, although the actual transcripts were not returned to the participants, member checking was conducted and a summary of the study results was shared to facilitate credibility of findings and trustworthiness. Other types of triangulations were not performed (e.g., investigator, theory, data source) [65] but method triangulation was done particularly in the area of pain relief.

## 6. Conclusions

This study emphasizes the importance of conducting qualitative research at the pre-RCT stage [19, 55, 56] to improve study intervention processes and help produce the best evidence for subsequent treatment and trials. We were able to evaluate our intervention content and delivery, trial design and conduct, study processes, and outcomes all aimed at improvement and refinement of future studies.

We found that vAPA was a feasible and effective self-management tool, allowing participants to assume an active role in their own pain management and allowing them to re-establish control over their pain. With a greater sense of control over pain, participants were further motivated to continue using APA to self-manage their pain. APA has a significant potential for providing a valuable public impact in decreasing the pain epidemic, opioid crisis, and healthcare utilization and costs.

## Figures and Tables

**Table 1:** Examples of participant responses coded under each categorized domain to evaluate feasibility of the vAPA.

*Acceptability (satisfaction, what participants like about intervention, intent to continue)*
(i) Noninvasive, I do not need to use medication.
(ii) It's a natural remedy, holistic, and this is helping to reduce the pain.
(iii) I like that it is non-pharmacologic, no side effects.
(iv) Like tiny meditation anytime the seeds are pressed, press during the higher levels of discomfort helps bring the intensity down because it gives something to focus on. I would continue because of the mediation effect, takes mind off of the pain; and will suggest to others.
(v) I would like to continue using APA for tingling in my feet.
(vi) I might try APA with my other pains (e.g., headache, etc.)
(vii) I referred to my brother-in-law. Since he started APA, he has not used any pain killers. My sister used it for sciatica pain and it worked immediately.

^*∗*^ *Usability and Implementation (participant engagement, recommendations)*
(i) Training videos were helpful especially first time, help as a guide to place the seeds.
(ii) Videos helpful, maybe add more information on videos for clarity on finding ear points.
(iii) I watched it a couple times to understand the process and how to locate the points.
(iv) Recommend to develop a website with these videos, tips, Q&As that anyone can access.
(v) Zoom sessions very helpful and informative in locating ear points, instructions were clear; had 2 zoom meetings, these were sufficient.
(vi) The Zoom session was very helpful, nice interaction, live responses.
(vii) Instructions and explain better in the beginning as to frequency/time for pressing, to press more frequently if needed for pain, and that this is not a cure but the best to have realistic expectations.
(viii) Pictures of ears really helped.
(ix) It might be helpful if there were more photo of the ear points.
(x) Would also be better if there is a bigger diagram of the ear, both ears.
(xi) I found that sending my ear photo and receiving feedback were helpful.
(xii) Nice to participate with social distancing.
(xiii) ^*∗*^Participant responses related to participant engagement as to *self-management and motivation in pain* are noted in Table 3.

*Practicality (cost, ability to carry out intervention)*
(i) I would recommend to others because you do not have to spend money, helps alleviate the pain wherever the pain is.
(ii) It [APA] is cost-effective.
(iii) I can find my own pressure points at any time in the comfort of my home instead of depending on having to go to the doctor.
(iv) It [APA] is easy, easy to apply treatment, seeds/tapes stayed on very well, easy to find ear points.
(v) Small seeds and tapes, not easily noticed by others. I do not have to go to therapist, the treatment is simple to use and I can use whenever I feel pain.
(vi) I did not have to go anywhere, can do it [APA] at home.
(vii) I do not have to go to doctor's office, able to do all online.
(viii) I did not have problems finding the ear points.

^*∗*^ *Perceived Benefits*
(i) Pain went from 7 to 4 = 30 to 40% improvement, very happy with this.
(ii) If push seeds, pain go down to 1, normally have pain at 5.
(iii) Pain is constant but able to get it down with pressing the seeds; there is a change and happy with change.
(iv) You can start feeling results almost immediately.
(v) Pain seems to recur a lot on days without seeds, pain is less frequent.
(vi) Back pain is better, numbness down the leg is still a challenge.
(vii) I experienced improvement on the numbness in my toe, can walk a little bit further, and increased physical activity.
(viii) Stopped tingling feeling in feet when seeds are pressed, reoccurrence of tingling is less by pressing the seeds.
(ix) I was not into alternative medicine initially but this helps control the anxiety of getting the intense pain.
(x) It [APA] relaxes, helps with pain and stress, gets mind off pain.
(xi) When I put on the seeds for the first time, I had the best sleep in years. Has been getting good sleep since. Also noticed I am more consistent with my daily exercise because I do not wake up with pain anymore.
(xii) It [APA] helped me sleep better.
(xiii) Sleep quality is better, do not wake up with pain.
(xiv) ^*∗*^Participant responses related to perceived benefits as *to better control of pain*, *less use of pain medications*, and *expectations for pain relief* are noted in Table 3.

*Potential Barriers*
(i) Hard to find pressure point to place APA, need someone help place the seeds.
(ii) Seeds and tape fall off at times.
(ii) Tapes are irritating, itchy, and sore sometimes.
(iv) Sore after pressing but soreness goes away, would rather have soreness on the ear from APA than have pain.
(v) Nothing.

**Table 2:** Demographic characteristics of the participants.

Variable	*N* (SD)
Age	
Mean (SD) (range)	52.39 (18.16) (24–80)

Gender (*n*)	
Male	5
Female	13

Body mass index (SD)	
Mean (SD) (range)	27.03 (4.53) (18.40–35.20)

Race/ethnicity (*n*)^*∗*^	
White	14
Black/African American	1
Others	2

Marital Status (*n*)	
Currently married/live with partner	10
Divorced	3
Widowed	1
Never married	4

Employment Situation (*n*)	
Working (full time)	8
Not employed	8
On leave	2

Education level (*n*)	
High school	1
Technical or vocational school	1
College	11
Graduate	5

Estimated income before taxes (*n*)	
$20,000 to $39,999	3
$40,000 to $59,000	3
$60,000 to $100,000	7
More than $100,000	5

Current prescribed pain medication	
Yes	10
No	8

Current prescribed sleep medication	
Yes	3
No	15

Current over the counter pain medication	
Yes	11
No	7

Current over the counter sleep medication	
Yes	1
No	17

^*∗*^ *n* varied due to missing data, SD = standard deviation.

**Table 3:** Examples of participant responses reflecting study themes.

^*∗*^ *vAPA is feasible*
(i) ^*∗*^Several participant sample responses are reflected in Table 1 reflecting acceptability, usability, practicality, and perceived benefits.

*Better control of pain*
(i) Being able to press the seeds when pain recurs is very convenient for me, because I can easily take care of my pain even when I am working without having to stop and take medication. I feel that it helps me stay positive and confident that I can manage my own pain without having to rely on meds.
(ii) Feel better control over pain especially when overdoing and gets a lot of pain, I press the seeds and get relief especially when pain is aggravated.
(iii) Better control, can press [ear points] anytime.
(iv) Have more control of pain, press the seeds when in pain and pain improves.
(v) Feel better control over pain though just realized recently that can press more if needed for pain, able to get it down with pressing the seeds.
(vi) Better control of tingling by pressing points.
(vii) Wake up from pain then press the seeds and then able to fall asleep.

*Less use of pain medications*
(i) I am using less pain medication. Usually takes aspirin, tramadol and muscle relaxant as needed. Only needed to take 1 muscle relaxant during the trial.
(ii) I still use tylenol but less.
(iii) Used to take ibuprofen but has not used any at all since APA.
(iv) Needed less ibuprofen.
(v) Most of the time I have not needed to take any pain medication.
(vi) Don't usually take meds but took tylenol 3000 mg in the past and ice packs, have not had to do these.
(vii) Reduced use of pain medications like ibuprofen, lidocaine, and less use of other natural remedies like CBD oil, massage, epsom salts.
(viii) Has not been to a provider for pain.

*Self-management and motivation in pain*
(i) Self-motivation is important, pain should be enough motivation, do not see anything else that could be done better to motivate [to do APA].
(ii) Motivation is a personal thing; the seeds have a positive effect.
(iii) I believe this treatment is self-motivating if the patient has faith in it and finds that it helps.
(iv) Pain relief was motivation enough.
(v) This is a really good way not to use drugs.
(vi) Since I am trying to avoid using pain medication and my pain comes and goes, the treatment is an alternative choice to manage my pain.
(vii) To avoid surgery, I can use APA to manage pain.

*Expectations for pain relief*
(i) Expect to get pain down to 3 or 4 from 8, she was getting this pain relief with the APA.
(ii) Pain is 4-5 average, do not want to be on the medication forever so this [APA] keeps mind off it; even a decrease to 2-3 pain is ok.
(iii) 1 point drop is ok, immediate effect is better but realistic that it will take a while.
(iv) Just a decrease of 1-2 points help, takes the edge off when seeds are pressed, couple hours relief and takes a little time for pain relief, about 15–30 minutes.
(v) Pain down to 2 and 3 is ok. Current average pain is 3–5 and if goes down to 2-3, this is my minimal expectation and this is being met.
(vi) Any program that helps the pain is good.

## Data Availability

Data are available on request.
